The article "Hepatitis C Virus Core Protein Down-Regulates p21Waf1/Cip1 and Inhibits Curcumin-Induced Apoptosis through MicroRNA-345 Targeting in Human Hepatoma Cells" was retracted in 2020. Reasons: duplicated images; unreliable results or conclusions; concerns about the data; concerns about the images.

# Hepatitis C Virus Core Protein Down-Regulates p21^Waf1/Cip1^ and Inhibits Curcumin-Induced Apoptosis through MicroRNA-345 Targeting in Human Hepatoma Cells

**DOI:** 10.1371/journal.pone.0061089

**Published:** 2013-04-08

**Authors:** Tzu-Yue Shiu, Shih-Ming Huang, Yu-Lueng Shih, Heng-Cheng Chu, Wei-Kuo Chang, Tsai-Yuan Hsieh

**Affiliations:** 1 Graduate Institute of Medical Sciences, National Defense Medical Center, Taipei, Taiwan, R.O.C.; 2 Division of Gastroenterology, Department of Internal Medicine, Tri-Service General Hospital, National Defense Medical Center, Taipei, Taiwan, R.O.C.; 3 Department of and Graduate Institute of Biochemistry, National Defense Medical Center, Taipei, Taiwan, R.O.C.; Kaohsiung Medical University Hospital, Kaohsiung Medical University, Taiwan

## Abstract

**Background:**

Hepatitis C virus (HCV) has been reported to regulate cellular microRNAs. The HCV core protein is considered to be a potential oncoprotein in HCV-related hepatocellular carcinoma, but HCV core-modulated cellular microRNAs are unknown. The HCV core protein regulates *p21^Waf1/Cip1^* expression. However, the mechanism of HCV core-associated *p21^Waf1/Cip1^* regulation remains to be further clarified. Therefore, we attempted to determine whether HCV core-modulated cellular microRNAs play an important role in regulating *p21^Waf1/Cip1^* expression in human hepatoma cells.

**Methods:**

Cellular microRNA profiling was investigated in core-overexpressing hepatoma cells using TaqMan low density array. Array data were further confirmed by TaqMan real-time qPCR for single microRNA in core-overexpressing and full-length HCV replicon-expressing cells. The target gene of microRNA was examined by reporter assay. The gene expression was determined by real-time qPCR and Western blotting. Apoptosis was examined by annexin V-FITC apoptosis assay. Cell cycle analysis was performed by propidium iodide staining. Cell proliferation was analyzed by MTT assay.

**Results:**

HCV core protein up- or down-regulated some cellular microRNAs in Huh7 cells. HCV core-induced microRNA-345 suppressed *p21^Waf1/Cip1^* gene expression through targeting its 3′ untranslated region in human hepatoma cells. Moreover, the core protein inhibited curcumin-induced apoptosis through p21^Waf1/Cip1^-targeting microRNA-345 in Huh7 cells.

**Conclusion and Significance:**

HCV core protein enhances the expression of microRNA-345 which then down-regulates *p21^Waf1/Cip1^* expression. It is the first time that HCV core protein has ever been shown to suppress *p21^Waf1/Cip1^* gene expression through miR-345 targeting.

## Introduction

Hepatitis C virus (HCV) infection is a major cause of chronic hepatitis, cirrhosis and hepatocellular carcinoma (HCC) [1]. The viral genome encodes a single polyprotein precursor of approximately 3000 amino acids, which is cleaved by cellular and viral proteases into three structural proteins (Core, E1, and E2) and seven nonstructural proteins (p7, NS2, NS3, NS4A, NS4B, NS5A, and NS5B) [2]. The HCV core protein, a component of the viral capsid, is initially split from the viral polyprotein between amino acid residues 191 and 192 by a signal peptidase within the endoplasmic reticulum (ER) lumen. Subsequently, this full-length core protein (amino acids 1–191, 191 a.a.) is further cleaved into a mature form (amino acids 1–173, 173 a.a.) by a signal peptide peptidase (SPP) [3], [4]. Further processing of the core protein in the C-terminal region produces a more truncated form, which can only be produced from limited HCV genotypes [5]. The full-length core protein localizes in the cytoplasm, whereas truncated core proteins (amino acids 1–173 and 1–151) localize in the nucleus [3], [5], [6]. Some cytoplasmic and nuclear proteins have been reported to interact with HCV core protein [7]–[10]. Recently, Moriishi *et al.* have reported that HCV core protein binds to the proteasome activator PA28γ in the nucleus, which induces liver steatosis and hepatocarcinogenesis through a PA28γ-dependent pathway in core transgenic mice [11], [12]. These studies suggest that HCV core as a regulatory protein may be involved in hepatocarcinogenesis during chronic HCV infection.

The article "Hepatitis C Virus Core Protein Down-Regulates p21Waf1/Cip1 and Inhibits Curcumin-Induced Apoptosis through MicroRNA-345 Targeting in Human Hepatoma Cells" was retracted in 2020. Reasons: duplicated images; unreliable results or conclusions; concerns about the data; concerns about the images.

MicroRNAs are small, endogenous non-coding RNA molecules that regulate the expression of at least one-third of human genes by inhibiting mRNA translation or inducing its degradation depending on the degree of complementarity [13], [14]. Studies have shown that cellular microRNAs play an important role in various physiological and pathological processes including human cancers [15], [16]. It has been reported that some cellular microRNAs are misregulated in HCV-related HCC [17], [18]. Recently, HCV-specific effects on the modulation of cellular microRNAs have been shown in full-length HCV genome-expressing HepG2 cells [19]. These studies suggest that HCV proteins-modulated microRNAs may function as oncogenes or as tumor suppressor genes.

The misregulation of *p21^Waf1/Cip1^* gene expression is frequently observed in human cancers [20]. Hepatocarcinogenesis requires continuous cellular stresses such as viral replication, oxidative stress, inflammation, and continued cell death after regeneration, to receive DNA damage in hepatocytes [1], [21]. The up-regulation of *p21^Waf1/Cip1^* gene expression by cellular stresses may prevent hepatocytes from transformation by inducing a sufficient G1 span to trigger apoptosis or repair DNA damage [20]. Although p21^Waf1/Cip1^ deficiency may not be sufficient to hepatocarcinogenesis, *p21^Waf1/Cip1^* gene misregulation may be involved in multistep hepatocarcinogenesis. Moreover, p21^Waf1/Cip1^ may be a target for cancer therapy [20]. Curcumin, a potential anticancer agent, has been used in preclinical in vitro and in vivo models of HCC [22]. Curcumin exerts its effect on anticancer, at least in part, by triggering apoptosis. Curcumin may induce apoptosis through p21^Waf1/Cip1^-dependent pathway [23]. Recently, curcumin has been reported to induce apoptosis in human hepatoma cell lines [24].

The article "Hepatitis C Virus Core Protein Down-Regulates p21Waf1/Cip1 and Inhibits Curcumin-Induced Apoptosis through MicroRNA-345 Targeting in Human Hepatoma Cells" was retracted in 2020. Reasons: duplicated images; unreliable results or conclusions; concerns about the data; concerns about the images.

The HCV core protein is considered to be involved in hepatocarcinogenesis [11], [12], [25]. HCV has been reported to regulate cellular microRNAs [19]. Moreover, the core protein can regulate p21^Waf1/Cip1^ expression [26]–[29]. In this study, we analyzed the expression profiles of cellular microRNAs in core-overexpressing human hepatoma cells compared to cells nonexpressing core. The HCV core protein was able to up-regulate microRNA-345 (miR-345) expression in human hepatoma cells. The HCV core-induced miR-345 suppressed endogenous *p21^Waf1/Cip1^* gene expression through targeting its 3′ untranslated region (3′UTR) in HepG2 cells and curcumin-stimulated Huh7 cells. In addition, the core protein inhibited curcumin-induced apoptosis through p21^Waf1/Cip1^-targeting miR-345 in Huh7 cells.

## Materials and Methods

### Antibodies, MicroRNA mimics, Mutant microRNA mimic, Small interfering RNA, MicroRNA inhibitor, and Chemicals

Anti-HA epitope antibody (catalog no. 11583816001) was purchased from Roche Applied Science, anti-p21^Waf1/Cip1^ antibody (catalog no. sc-6246) was from Santa Cruz Biotechnology, and anti-β-actin antibody (catalog no. A1978) was from Sigma-Aldrich. Anti-HCV core (catalog no. ab2740) and anti-HCV NS5B (catalog no. ab35586) antibodies were purchased from Abcam. Human microRNA-345 (hsa-miR-345, MIMAT0000772) and microRNA-93 (hsa-miR-93, MIMAT0000093) mimics were purchased from Thermo Scientific. Mutant microRNA-345 mimic was synthesized by Thermo Scientific. The sequence was 5′- GCUCUGACCUAGUCCAGGGCUC-3′. The four mutated sites are underlined. Human p21^Waf1/Cip1^ small interfering RNA (siRNA, catalog no. sc-29427) was purchased from Santa Cruz Biotechnology. Human miR-345 inhibitor (MH12733) was purchased from Applied Biosystems. Curcumin (catalog no. C7727) and dimethyl sulfoxide (DMSO, catalog no. D2650) were purchased from Sigma-Aldrich. Curcumin was dissolved in DMSO to 100 mM and stored at −20°C until use.

### Plasmid Construction

Plasmid pT-REx-HA-Core was generated by cloning the N-terminus HA-tagged HCV core coding sequence (genotype 1b strain) [30] into pT-REx-DEST30 vector (Invitrogen) according to the manufacturer's instructions. HA-Core was amplified by PCR using pcDNA3-HA-Core191 (amino acids 1–191) as a template. Primers used for cloning HA-Core191 were forward 5′-ACCATGTATCCATATGATGT-3′ and reverse 5′-TCAAGCGGAAGCTGGGATGG-3′. Primers used for cloning HA-Core173 (amino acids 1–173) were forward 5′-ACCATGTATCCATATGATGT-3′ and reverse 5′-TCAAGAGCAACCGGGCAGAT-3′. Primers used for cloning HA-Core153 (amino acids 1–153) were forward 5′-ACCATGTATCCATATGATGT-3′ and reverse 5′-TCAATGTGCCAGGGCTCTGG-3′. A control vector, pT-REx-Mock, was created by deleting HCV core coding sequence from the above construct using BsrGI restriction enzyme. Wild-type human *p21^Waf1/Cip1^* 3′UTR was amplified by PCR from human genomic DNA and cloned into pGL3-Control vector (Promega) immediately downstream of luciferase reporter gene but upstream of poly (A) signal using XbaI restriction enzyme to generate pGL3-Control-p21 3′UTR Sense (S) and pGL3-Control-p21 3′UTR Antisense (AS) vectors. Primers used for cloning human *p21^Waf1/Cip1^* 3′UTR were forward 5′-CCCTCTAGATCCGCCCACAGGAAGCCTGC-3′ and reverse 5′-CCCTCTAGAAAAGTCACTAAGAATCATTT-3′. The XbaI site is underlined. The mutant *p21^Waf1/Cip1^* 3′UTR in the seed sequence of hsa-miR-345 was generated by PCR and ligation of two pieces of DNA fragments, and then cloned into pGL3-Control vector to yield a pGL3-Control-p21 3′UTR Mutant vector. Primer pairs used for cloning mutated *p21^Waf1/Cip1^* 3′UTR were forward 5′-CCCTCTAGATCCGCCCACAGGAA-3′ and reverse 5′-CCTTGTTCCGCTGCTAATCA-3′, and were forward 5′-TCAGAGACATTTTAAGATGGTGGC-3′ and reverse 5′-CCCTCTAGAAAAGTCACTAAGAA-3′. The XbaI site is underlined.

The article "Hepatitis C Virus Core Protein Down-Regulates p21Waf1/Cip1 and Inhibits Curcumin-Induced Apoptosis through MicroRNA-345 Targeting in Human Hepatoma Cells" was retracted in 2020. Reasons: duplicated images; unreliable results or conclusions; concerns about the data; concerns about the images.

### Full-length HCV Replicon

A genotype 1b strain of full-length HCV replicon (HCV-N) [31] was kindly provided by Dr. Michael M.C. Lai at Institute of Molecular Biology, Academia Sinica, Taipei, Taiwan, R.O.C.. A control replicon HCV-A357T, which expresses only the initial five amino acids of the core protein due to introduction of a termination codon, was created by the change of one nucleotide at HCV nt 357 in pHCV-N (Fig. 1D, upper panel) using QuikChange Lightning Site-Directed Mutagenesis Kit (Agilent Technologies) according to the manufacturer's instructions.

**Figure 1:** HCV core protein up-regulates miR-345 and miR-93 expression in human hepatoma cells. (**A**) Huh7 cells were transiently transfected with empty vector (labeled with Mock) and three HCV core gene-expressing vectors, pT-REx-HA-Core191 (labeled with HA-Core191), pT-REx-HA-Core173 (labeled with HA-Core173), and pT-REx-HA-Core153 (labeled with HA-Core153), for core protein with amino acids 1–191, 1–173 and 1–153, respectively. At 48 hours after transfection, the expression of HCV core protein was analyzed by immunoprecipitation. (**B**) Huh7 cells were transiently transfected with empty vector and two HCV core gene-expressing vectors, pT-REx-HA-Core191, and pT-REx-HA-Core173, for core protein with amino acids 1–191 and 1–173, respectively. At 48 hours after transfection, cellular microRNA profiling was analyzed by TaqMan low density array. Three microRNAs, miR-21, miR-345 and miR93, of thirty-one microRNAs were indicated. (**C**) Huh7 and HepG2 cells were transiently transfected with empty vector (labeled with Mock) and three HCV core gene-expressing vectors, pT-REx-HA-Core191 (labeled with HA-Core191), pT-REx-HA-Core173 (labeled with HA-Core173), and pT-REx-HA-Core153 (labeled with HA-Core153), for core protein with amino acids 1–191, 1–173 and 1–153, respectively. At 48 hours after transfection, relative expression of miR-345 or miR-93 was determined by TaqMan real-time qPCR in Huh7 cells (left upper panel) and HepG2 cells (right upper panel). The expression of HCV core protein was analyzed by Western blotting (left lower and right lower panels). (**D**) The genotype 1b strain of full-length HCV replicon (HCV-N) and control replicon HCV-A357T which expresses only the initial five amino acids of the core protein due to introduction of a termination codon, was created by the change of one nucleotide at HCV nt 357 in pHCV-N (upper panel). HCV core and NS5B gene expression in full-length HCV replicon-expressing cells was analyzed by immunoprecipitation followed by Western blotting and Western blotting only respectively (left lower panel). The relative expressions of miR-345 and miR-93 were determined by TaqMan real-time qPCR in full-length HCV replicon-expressing Huh7 cells (right lower panel). Data was shown as the means ± S.D. from triplicate experiments. *P<0.05, **P<0.001.

### In Vitro Transcription of HCV RNA

pHCV-N DNA was linearized with XbaI, purified by phenol/chloroform extraction and ethanol precipitation [31], and then the linearized DNA was used as template to transcribe full-length HCV RNA using Riboprobe in vitro Transcription Systems (Promega, catalog no. P1440) following the manufacturer's protocol. The integrity of RNA transcripts was determined by agarose gel electrophoresis and ethidium bromide staining.

### Cell Culture and Transfection

Human hepatoma cell lines, Huh7 and HepG2 cells, were cultured at 37°C in a humidified incubator containing 5% CO_2_ in Dulbecco's modified Eagle's medium supplemented with 10% heat-inactivated fetal bovine serum (Hyclone). Plasmid DNA was transfected into cells using GenJet In Vitro DNA Transfection Reagent Ver. II (SignaGen Laboratories) following the manufacturer's protocol. To establish the full-length HCV replicon-expressing system in Huh7 cells, HCV RNA was transfected into cells using TransIT-mRNA Transfection Kit (Mirus Bio LLC) according to the manufacturer's instructions. The siRNA, microRNA mimic and inhibitor were transfected into cells using GenMute siRNA & DNA Transfection Reagent (SignaGen Laboratories) following the manufacturer's protocol.

The article "Hepatitis C Virus Core Protein Down-Regulates p21Waf1/Cip1 and Inhibits Curcumin-Induced Apoptosis through MicroRNA-345 Targeting in Human Hepatoma Cells" was retracted in 2020. Reasons: duplicated images; unreliable results or conclusions; concerns about the data; concerns about the images.

### RNA Extraction

Total RNA was extracted using miRNeasy Mini Kit (Qiagen) according to the manufacturer's protocol. The trace quantities of genomic DNA were further removed using Turbo DNA-free Kit (Applied Biosystems) following the manufacturer's instructions.

### TaqMan Low Density Array for MicroRNA

TaqMan low density array was performed using Applied Biosystems 7900HT Fast Real-Time PCR System according to the manufacturer's protocol. Briefly, cDNA templates were synthesized using TaqMan MicroRNA Megaplex RT Kit (Applied Biosystems) following the manufacturer's instructions. A total reaction mixture containing RT products and TaqMan Universal PCR Master Mix (Applied Biosystems) was added to each line of TaqMan low density array card after gentle vortex mixing. Thermal cycler conditions were as follows: 50°C for 2 minutes, 94.5°C for 10 minutes, and then 40 cycles of 97°C for 30 seconds and 59.7°C for 1 minute. Cycle threshold was automatically given by SDS software v2.2 (Applied Biosystems) using automatic baseline settings and a threshold of 0.2. MammU6 was used as an internal control to normalize the amount of individual microRNA in each sample. Significant difference of relative microRNA expression was determined using the 2^−ΔΔCt^ method [32].

### TaqMan Real-time qPCR for Single MicroRNA Assay

cDNA template for single microRNA was synthesized using TaqMan MicroRNA RT Kit (Applied Biosystems) according to the manufacturer's protocol. Expression of specific microRNA was determined by real-time qPCR using TaqMan MicroRNA qPCR Kit (Applied Biosystems) following the manufacturer's instructions. MammU6 was used as an internal control to normalize the amount of specific microRNA in each sample. Significant difference of relative microRNA expression was determined as described above.

### Real-time qPCR

cDNA template was synthesized using ImProm-II Reverse Transcription System (Promega) according to the manufacturer's protocol. Expression of human p21^Waf1/Cip1^ mRNA was determined by real-time qPCR using Power SYBR Green PCR Master Mix (Applied Biosystems) following the manufacturer's instructions. The β-actin mRNA was used as an internal control to normalize the amount of human p21^Waf1/Cip1^ mRNA in each sample. Primer sequences for human p21^Waf1/Cip1^ and β-actin mRNAs were described previously [33]. Significant difference of relative gene expression was determined as described above.

The article "Hepatitis C Virus Core Protein Down-Regulates p21Waf1/Cip1 and Inhibits Curcumin-Induced Apoptosis through MicroRNA-345 Targeting in Human Hepatoma Cells" was retracted in 2020. Reasons: duplicated images; unreliable results or conclusions; concerns about the data; concerns about the images.

### Luciferase Reporter Assay

Cells were transfected with luciferase reporter vector in combination with microRNA mimic. All transfections included pRL-TK vector (Promega) for normalization. Luciferase activity was analyzed by Dual-Glo Luciferase Assay System (Promega) according to the manufacturer's instructions. Renilla luminescence, expressed from pRL-TK vector, was used as an internal control to normalize the luciferase activity.

### Immunoprecipitation

Cell lysates were extracted using RIPA buffer (Sigma-Aldrich) supplemented with Halt Protease Inhibitor Cocktail (Thermo Scientific). The supernatants were incubated for 2 hours at 4°C with anti-HA epitope or anti-HCV core antibody, and then overnight at 4°C with Protein A-agarose beads (Roche Applied Science, catalog no. 11719408001). Following four washes with RIPA buffer, proteins were eluted for 10 minutes at 100°C with 2× Laemmli sample buffer (Sigma-Aldrich), electrophoresed on SDS-PAGE and electroblotted onto PVDF membranes (Millipore).

### Western Blotting

Cell lysates were extracted as described above. Cell lysates were electrophoresed on SDS-PAGE and electroblotted onto PVDF membranes. Anti-HA epitope, anti-HCV core, anti-HCV NS5B, anti-p21^Waf1/Cip1^, and anti-β-actin antibodies were used in Western blotting according to the manufacturer's protocol. β-actin was used as an internal control. Relative protein expression was quantified by BioSpectrum Imaging System (UVP).

### DNA Fragmentation Analysis

Genomic DNA from cells was extracted using Wizard Genomic DNA Purification Kit (Promega) according to the manufacturer's instructions. DNA ladder was determined by agarose gel electrophoresis and ethidium bromide staining.

### Annexin V-FITC Apoptosis Assay

Apoptotic cells were detected and quantified by fluorescence microscopy and FACS Calibur (Becton Dickinson) respectively, using Annexin V-FITC Apoptosis Detection Kit (BioVision) following the manufacturer's protocol.

### Cell Cycle Analysis

Cells were subjected to serum starvation for 24 hours to arrest cell growth, and then cultured in fresh serum-containing medium for 24 hours for cell cycle re-entry. Cells were harvested after trypsinization in serum-containing medium, centrifuged and suspended in phosphate buffered saline (PBS). The absolute ethanol was added drop-wise and cells were maintained overnight at −20°C to complete fixation. Cells were centrifuged, resuspended in PBS plus RNase A and propidium iodide (Sigma-Aldrich), and incubated at 37°C for 30 minutes. Fluorescence was measured and analyzed by FACS Calibur.

The article "Hepatitis C Virus Core Protein Down-Regulates p21Waf1/Cip1 and Inhibits Curcumin-Induced Apoptosis through MicroRNA-345 Targeting in Human Hepatoma Cells" was retracted in 2020. Reasons: duplicated images; unreliable results or conclusions; concerns about the data; concerns about the images.

### Cell Proliferation Assay (MTT assay)

Cell proliferation was determined using CellTiter 96 Non-Radioactive Cell Proliferation Assay (Promega) according to the manufacturer's instructions. To analyze cell proliferation, Huh7 cells were seeded in 96-well culture plates at 3000 cells per well. After 24 hours, the medium was replaced with fresh medium supplemented with increased amount of curcumin. At 24 hours after treatment, Dye Solution was added to each well and cells were incubated at 37°C for 2 hours. Solubilization/Stop Solution was then added to each well and the absorbance was measured at 570 nm using an ELISA reader. Relative cell number was calculated by normalizing the absorbance to untreated cells. Relative cell viability was compared to untreated cells.

### Statistical Analysis

Data was shown as the means ± SD from triplicate experiments. The two-sided Student's *t*-test was used for comparisons between experimental groups. *P*<0.05 was considered statistically significant.

## Results

### MicroRNA-345 and microRNA-93 are overexpressed in HCV core-overexpressing human hepatoma cells

It has been reported that the full-length HCV core protein (amino acids 1–191) is further cleaved into truncated forms (amino acids 1–173 and 1–153) [3], [5]. Although the truncated core protein localizes in the nucleus [3], [5], [6], only a small quantity of the core protein localizes to the nuclei of hepatocytes in chronically HCV-infected patients and core transgenic mice [25], [34], [35]. In this study, three core gene-expressing vectors for core protein with amino acids 1–191, 1–173 and 1–153, respectively, were transfected into Huh7 cells. Immunoprecipitation followed by Western blotting was used to determine HCV core expression. The results showed that three forms of HCV core protein were overexpressed in Huh7 cells (Fig. 1A). Interestingly, a small quantity of a product with lower molecule weight was observed when the full-length core gene was overexpressed in Huh7 cells (Fig. 1A, lane 2). This product may suggest a truncated core protein trimmed at the C-terminal region due to the intracellular processing of the full-length core protein. To investigate the effect of the full-length and mature core proteins on the modulation of cellular microRNAs, two core gene-expressing vectors for core protein with amino acids 1–191 and 1–173, respectively, were transfected into Huh7 cells, and then the expression profiles of cellular microRNAs was determined by TaqMan low density array at 48 hours after transfection. The result showed that thirty-one microRNAs exhibited a greater than 2-fold up- or down-regulation in full-length core (191 a.a.) or mature core (173 a.a.)-overexpressing Huh7 cells compared to cells nonexpressing core (Fig. 1B). The HCV core protein can regulate p21^Waf1/Cip1^ expression [26]–[29]. Recently, Wu *et al.* have reported that human *p21^Waf1/Cip1^* gene expression can be inhibited by twenty-eight microRNAs in HEK 293 cells [33]. In this study, we indicated that two p21^Waf1/Cip1^-targeting microRNAs, microRNA-345 (miR-345) and microRNA-93 (miR-93), were up-regulated in core-overexpressing Huh7 cells (Fig. 1B). Array data were further confirmed by TaqMan real-time qPCR for miR-345 and miR-93 in Huh7 and HepG2 cells. Three core gene-expressing vectors for core protein with amino acids 1–191, 1–173 and 1–153, respectively, were transfected into cells, and then the relative expression of miR-345 and miR-93 was determined at 48 hours after transfection. The results showed that miR-345 and miR-93 were overexpressed with more than 3.5- and 2-fold changes, respectively, in mature core (173 a.a.) and more truncated core (153 a.a.)-overexpressing Huh7 cells but not in full-length core (191 a.a.)-overexpressing cells compared to cells nonexpressing core (Fig. 1C, left upper panel). Similar results also indicated in mature core and more truncated core-overexpressing HepG2 cells but not in full-length core-overexpressing cells (Fig. 1C, right upper panel).

The article "Hepatitis C Virus Core Protein Down-Regulates p21Waf1/Cip1 and Inhibits Curcumin-Induced Apoptosis through MicroRNA-345 Targeting in Human Hepatoma Cells" was retracted in 2020. Reasons: duplicated images; unreliable results or conclusions; concerns about the data; concerns about the images.

To further verify the expressions of cellular microRNAs in full-length HCV replicon-expressing system, the full-length HCV replicon was transfected into Huh7 cells. At 96 hours after transfection, immunoprecipitation followed by Western blotting was used to determine HCV core expression, and Western blotting only for NS5B expression (Fig. 1D, left lower panel, lane 2). The relative expressions of miR-345 and miR-93 were determined by TaqMan real-time qPCR. The results showed that miR-345 induction was not significantly affected in full-length HCV replicon-expressing system in Huh7 cells compared to control cells and untreated cells (Fig. 1D, right lower panel, third bar pair). Indeed, there is no detectable or little, if any, amount of truncated form of HCV core protein expression in full-length HCV replicon-expressing system in Huh7 cells (Fig. 1D, left lower panel, lane 2). Furthermore, miR-93 overexpression in full-length HCV replicon-expressing cells but not in full-length core-overexpressing cells suggested that other HCV proteins might up-regulate miR-93 expression. Together, these results demonstrate that truncated HCV core proteins (amino acids 1–173 and 1–153) up-regulate cellular miR-345 and miR-93 expression in human hepatoma cells.

The article "Hepatitis C Virus Core Protein Down-Regulates p21Waf1/Cip1 and Inhibits Curcumin-Induced Apoptosis through MicroRNA-345 Targeting in Human Hepatoma Cells" was retracted in 2020. Reasons: duplicated images; unreliable results or conclusions; concerns about the data; concerns about the images.

### MicroRNA-345 down-regulates *p21^Waf1/Cip1^* gene expression in human hepatoma cells

It has been reported that human *p21^Waf1/Cip1^* gene expression can be inhibited by miR-345 and miR-93 in HEK 293 cells [33]. Because the different cell types might generate different results, the effects of miR-345 and miR-93 on human *p21^Waf1/Cip1^* gene expression were examined in human hepatoma cells. Two luciferase reporter vectors which bear the sense and antisense 3′UTRs from human *p21^Waf1/Cip1^* gene, respectively, were used in luciferase reporter assay (Fig. 2A, upper panel). The relative luciferase activity was determined in Huh7 and HepG2 cells at 24 hours after transfection. The results showed that the treatment with miR-345 mimic led to a significant reduction of luciferase activity in p21 3′UTR Sense construct-transfected Huh7 cells, but treatment with miR-93 mimic had no significant inhibition in luciferase activity (Fig. 2A, left lower panel, second bar cluster). Moreover, treatment with a mixture of miR-345 and miR-93 mimics also had no double reduction of luciferase activity (Fig. 2A, left lower panel, second bar cluster). As expected, miR-345 and miR-93 mimics had no effect in control vector-transfected and p21 3′UTR Antisense construct-transfected Huh7 cells (Fig. 2A, left lower panel, first and third bar clusters). Similar results also indicated in HepG2 cells (Fig. 2A, right lower panel). We further examined human *p21^Waf1/Cip1^* gene expression at protein level when miR-93 mimic was transfected into HepG2 cells. As the results in luciferase reporter assay (Fig. 2A, left lower and right lower panels), *p21^Waf1/Cip1^* expression at protein level was not suppressed by miR-93 in HepG2 cells (Fig. S1). These results demonstrated that human *p21^Waf1/Cip1^* gene may be not a target of miR-93 in human hepatoma cells. We further focused on miR-345 to identify the seed sequence in human *p21^Waf1/Cip1^* 3′UTR by using computational tools, miRanda (http://www.microrna.org/microrna/home.do) and TargetScan (http://www.targetscan.org/) (Fig. 2B, left panel). To further verify the seed sequence of miR-345, two luciferase reporter vectors which bear the wild-type and mutant (mutated in the seed sequence of miR-345) 3′UTRs from human *p21^Waf1/Cip1^* gene, respectively, were used in luciferase reporter assay (Fig. 2B, left panel, mutated sites are underlined). The results showed that wild-type miR-345 mimic can significantly inhibit the luciferase activity in wild-type p21 3′UTR construct-transfected Huh7 cells but not in mutant p21 3′UTR construct-transfected cells (Fig. 2B, right panel, second and third bar pairs). However, an additional experiment with mutant miR-345 mimic (Fig. 2B, left panel, mutated sites are underlined) and mutant p21 3′UTR with restoring complementarity was able to show a significant inhibition of luciferase activity (Fig. 2B, right panel, fourth bar pair). These results showed that miR-345 may down-regulate human *p21^Waf1/Cip1^* gene expression through targeting its 3′UTR in human hepatoma cells. To further verify the down-regulation of endogenous *p21^Waf1/Cip1^* gene expression by miR-345, p21^Waf1/Cip1^ mRNA and protein levels were examined in HepG2 cells at 24 hours after transfection with miR-345 mimic. As expected, *p21^Waf1/Cip1^* gene expression at mRNA and protein levels was suppressed with the increased amount of miR-345 mimic in HepG2 cells (Fig. 2C, left and right panels). Together, these results demonstrate that miR-345 down-regulates *p21^Waf1/Cip1^* gene expression through targeting its 3′UTR in human hepatoma cells.

The article "Hepatitis C Virus Core Protein Down-Regulates p21Waf1/Cip1 and Inhibits Curcumin-Induced Apoptosis through MicroRNA-345 Targeting in Human Hepatoma Cells" was retracted in 2020. Reasons: duplicated images; unreliable results or conclusions; concerns about the data; concerns about the images.

**Figure 2:** MicroRNA-345 down-regulates *p21^Waf1/Cip1^* gene expression through targeting its 3′UTR but not microRNA-93 in human hepatoma cells. (**A**) Two luciferase reporter vectors, pGL3-Control-p21 3′UTR Sense (S) and pGL3-Control-p21 3′UTR Antisense (AS) which bear the sense and antisense 3′UTRs from human *p21^Waf1/Cip1^* gene, respectively, were constructed (upper panel). Huh7 cells and HepG2 cells were transfected with p21 3′UTR sense or antisense luciferase reporter vector in combination with miR-345 mimic, miR-93 mimic or a mixture of miR-345 and miR-93 mimics. At 24 hours after transfection, Huh7 cells (left lower panel) and HepG2 cells (right lower panel) were collected for luciferase reporter assay. (**B**) Base-pairing between mature hsa-miR-345 and target site in human *p21^Waf1/Cip1^* 3′UTR is shown (left panel). One luciferase reporter vector, pGL3-Control-p21 3′UTR Mutant (mutated in the seed sequence of miR-345), was constructed. Mutant miR-345 mimic was synthesized. The mutated site is underlined (left panel). Huh7 cells were transfected with wild-type p21 3′UTR sense or mutant p21 3′UTR luciferase reporter vector in combination with wild-type or mutant miR-345 mimic. At 24 hours after transfection, Huh7 cells were collected for luciferase reporter assay. The experiment with mutant miR-345 mimic and mutant p21 3′UTR with restoring complementarity was performed (right panel). (**C**) HepG2 cells were transiently transfected with the increased amount of miR-345 mimic for 24 hours. The *p21^Waf1/Cip1^* gene expression was analyzed by real-time qPCR (left panel) and Western blotting (right panel). β-actin served as an internal control. Data was shown as the means ± S.D. from triplicate experiments. *P<0.05.

The article "Hepatitis C Virus Core Protein Down-Regulates p21Waf1/Cip1 and Inhibits Curcumin-Induced Apoptosis through MicroRNA-345 Targeting in Human Hepatoma Cells" was retracted in 2020. Reasons: duplicated images; unreliable results or conclusions; concerns about the data; concerns about the images.

### MicroRNA-345 inhibits curcumin-induced apoptosis through down-regulation of *p21^Waf1/Cip1^* gene expression in Huh7 cells

Curcumin, a potential anticancer agent, has been used in preclinical in vitro and in vivo models of HCC [22]. Recently, curcumin has been reported to induce apoptosis in Huh7 cells [24]. In this study, we showed that *p21^Waf1/Cip1^* gene expression at protein level was enhanced with increased amount of curcumin in Huh7 cells (Fig. 3A, upper panel). To investigate the functional relevance of *p21^Waf1/Cip1^* up-regulation and curcumin treatment in Huh7 cells, annexin V-FITC apoptosis assay, MTT assay, and cell cycle analysis were performed. The results showed that curcumin induced apoptosis and inhibited cell viability in Huh7 cells in a dose-dependent manner (Fig. 3A, middle and left lower panels). Furthermore, the result also showed that S-phase entry of cell cycle was slightly inhibited in Huh7 cells in response to high doses of curcumin (Fig. 3A, right lower panel). To further verify that the up-regulation of *p21^Waf1/Cip1^* gene expression involved in curcumin-induced apoptosis in Huh7 cells, curcumin-stimulated cells were transfected with increased amount of p21^Waf1/Cip1^ siRNA, and then apoptosis was analyzed by using DNA fragmentation analysis at 24 hours after transfection. The result showed that apoptosis was inhibited as presented in DNA ladder disappeared when *p21^Waf1/Cip1^* gene expression at protein level was suppressed in curcumin-stimulated Huh7 cells (Fig. 3B), indicating that curcumin induced apoptosis through up-regulation of *p21^Waf1/Cip1^* gene expression in Huh7 cells. Similar results were also showed in Figure 3C. Curcumin had no effect on the modulation of cellular miR-345 expression in Huh7 cells (Fig. S2). As expected, *p21^Waf1/Cip1^* gene expression at protein level was suppressed by miR-345 mimic in curcumin-stimulated Huh7 cells in a dose-dependent manner (Fig. 3C, upper panel). Curcumin-induced apoptosis was inhibited with increased amount of miR-345 mimic (Fig. 3C, left middle panel). Moreover, the introduction of miR-345 mimic enhanced cell viability in curcumin-stimulated Huh7 cells (Fig. 3C, right middle panel). The number of apoptotic cells (early and late apoptotic cells) had a maximum reduction of about 55% when curcumin-stimulated cells were transfected with 50 nM miR-345 mimic (Fig. 3C, left lower and right lower panels). In HepG2 cells, we also showed that curcumin induced apoptosis, but curcumin had no effect on the modulation of *p21^Waf1/Cip1^* gene expression. The results indicated that curcumin was able to induce apoptosis through a p21^Waf1/Cip1^-independent pathway in HepG2 cells (Fig. S4). Together, these results demonstrate that miR-345 inhibits curcumin-induced apoptosis through down-regulation of *p21^Waf1/Cip1^* gene expression in Huh7 cells.

The article "Hepatitis C Virus Core Protein Down-Regulates p21Waf1/Cip1 and Inhibits Curcumin-Induced Apoptosis through MicroRNA-345 Targeting in Human Hepatoma Cells" was retracted in 2020. Reasons: duplicated images; unreliable results or conclusions; concerns about the data; concerns about the images.

**Figure 3:** MicroRNA-345 inhibits curcumin-mediated apoptosis through down-regulation of *p21^Waf1/Cip1^* gene expression in Huh7 cells. (**A**) Huh7 cells were treated with different doses (6.25, 12.5, 25 and 50 µM) of curcumin for 24 hours. DMSO served as control (labeled with 0 µM). The *p21^Waf1/Cip1^* gene expression at protein level was determined by Western blotting (upper panel). β-actin served as an internal control. Apoptosis was determined by annexin V-FITC apoptosis assay (middle panel). Cell proliferation was analyzed by MTT assay (left lower panel). Cell cycle distribution was examined by cell cycle analysis (right lower panel). (**B**) Huh7 cells were transfected with the increased amount of *p21^Waf1/Cip1^* siRNA in response to curcumin stimulation (50 µM) for 24 hours. Apoptosis was analyzed by DNA fragmentation analysis. The *p21^Waf1/Cip1^* gene expression at protein level was examined by Western blotting. (**C**) Huh7 cells were transfected with the increased amount of miR-345 mimic in response to curcumin stimulation (50 µM) for 24 hours. The *p21^Waf1/Cip1^* gene expression at protein level was examined by Western blotting (upper panel). β-actin served as an internal control. Apoptosis was analyzed by fluorescence microscopy (left middle panel) and FACS Calibur (left lower and right lower panels) using Annexin V-FITC apoptosis assay. Original magnifications ×200. Cells from early apoptotic stage were stained with annexin V-FITC, and appeared green. Cells from late apoptotic stage were stained with both annexin V-FITC and PI, and merged to be yellow. Cell proliferation was analyzed by MTT assay (right middle panel). Data was shown as the means ± S.D. from triplicate experiments. *P<0.05, **P<0.001.

### HCV core-induced microRNA-345 inhibits *p21^Waf1/Cip1^* gene expression in HepG2 cells and curcumin-stimulated Huh7 cells

It has been reported that the mature form (amino acids 1–173) of HCV core protein in the nucleus suppresses *p21^Waf1/Cip1^* gene expression in HepG2 cells [27]. To determine that HCV core-induced miR-345 down-regulated endogenous *p21^Waf1/Cip1^* gene expression, core expressing HepG2 cells were transfected with or without miR-345 inhibitor, and then *p21^Waf1/Cip1^* gene expression at protein level was determined at 24 hours after transfection. As expected, the mature form (amino acids 1–173) of the core protein suppressed *p21^Waf1/Cip1^* gene expression (Fig. 4A, lane 3). However, the suppression of *p21^Waf1/Cip1^* gene expression was attenuated in the presence of increased amount of miR-345 inhibitor (Fig. 4A, lane 3, lane 6 and lane 7). The full-length core protein (amino acids 1–191) slightly suppressed *p21^Waf1/Cip1^* gene expression (Fig. 4A, lane 2), this result may be due to the expression of a small quantity of the truncated core protein (Fig. 1A, lane 2). We have shown that only little amount of p21^Waf1/Cip1^ protein can be detected in Huh7 cells (Fig. 3A, upper panel, lane 1). Therefore, curcumin was used to induce endogenous *p21^Waf1/Cip1^* gene expression to investigate the inhibition of *p21^Waf1/Cip1^* gene expression by HCV-core-induced miR-345 in Huh7 cells. Similar results were also showed in Figure 4B. As expected, the mature form (amino acids 1–173) of the core protein suppressed *p21^Waf1/Cip1^* gene expression in curcumin-stimulated Huh7 cells (Fig. 4B, upper panel, lane 3). Similarly, the suppression of *p21^Waf1/Cip1^* gene expression was attenuated when mature core-expressing cells were transfected with miR-345 inhibitor (Fig. 4B, upper panel, lane 3, lane 6 and lane 7). Additionally, the suppression of curcumin-induced apoptosis by mature core protein (amino acids 1–173) was significantly attenuated in the presence of increased amount of miR-345 inhibitor (Fig. 4B, middle and lower panels). Together, these results demonstrate that HCV core-induced miR-345 inhibits endogenous *p21^Waf1/Cip1^* gene expression in HepG2 cells and curcumin-stimulated Huh7 cells.

The article "Hepatitis C Virus Core Protein Down-Regulates p21Waf1/Cip1 and Inhibits Curcumin-Induced Apoptosis through MicroRNA-345 Targeting in Human Hepatoma Cells" was retracted in 2020. Reasons: duplicated images; unreliable results or conclusions; concerns about the data; concerns about the images.

**Figure 4:** HCV core-induced microRNA-345 inhibits *p21^Waf1/Cip1^* gene expression in HepG2 cells and curcumin-stimulated Huh7 cells. (**A**) HCV core (amino acid 1–191 or 1–173)-expressing HepG2 cells were transfected with miR-345 inhibitor (5 nM or 10 nM). At 24 hours after transfection, *p21^Waf1/Cip1^* gene expression at protein level was analyzed by Western blotting. β-actin served as an internal control. (**B**) HCV core (amino acid 1–191 or 1–173)-expressing Huh7 cells in response to curcumin stimulation were transfected with miR-345 inhibitor (5 nM or 10 nM). At 24 hours after transfection, *p21^Waf1/Cip1^* gene expression at protein level was analyzed by Western blotting. β-actin served as an internal control (upper panel). Apoptosis was analyzed by fluorescence microscopy (middle panel) and FACS Calibur (lower panel) using Annexin V-FITC apoptosis assay. Original magnifications ×200. Cells from early apoptotic stage were stained with annexin V-FITC, and appeared green. Cells from late apoptotic stage were stained with both annexin V-FITC and PI, and merged to be yellow. Data was shown as the means ± S.D. from triplicate experiments. *P<0.05, **P<0.001.

The article "Hepatitis C Virus Core Protein Down-Regulates p21Waf1/Cip1 and Inhibits Curcumin-Induced Apoptosis through MicroRNA-345 Targeting in Human Hepatoma Cells" was retracted in 2020. Reasons: duplicated images; unreliable results or conclusions; concerns about the data; concerns about the images.

## Discussion

In this study, we determine the effect of a mature HCV core protein on miR-345 induction in human hepatoma cells. Moreover, HCV core-induced miR-345 suppresses *p21^Waf1/Cip1^* gene expression in HepG2 cells, and inhibits curcumin-mediated apoptosis through down-regulation of *p21^Waf1/Cip1^* gene expression in Huh7 cells.

HCV core protein has an effect on cellular microRNA regulation. HCV core protein is initially separated from HCV polyprotein by a signal peptidase. The full-length core protein (amino acids 1–191) localizes in the cytoplasm, which mainly functions as a component of the viral capsid. HCV core protein is considered to play a crucial role in hepatocarcinogenesis [11], [12], [25]. Many studies have reported that HCV core protein can interact with cytoplasmic and nuclear proteins [7]–[10]. Chen *et al.* has shown that HCV core protein interacts with Dicer, an RNase enzyme that generates mature microRNAs, in the cytoplasm, and then inhibits the function of Dicer [36]. This inhibitive effect may contribute to HCV replication [37]. The mature form (amino acids 1–173) of HCV core protein cleaved by SPP, which lacks the 174–191 peptide for attachment to ER membrane, enables subcellular distribution of the core protein [3]–[6]. Unlike full-length core protein (amino acids 1–191), mature form (amino acids 1–173) has been reported to mainly localize to nucleus [3], [5], [6]. Some studies have shown that a small quantity of HCV core protein localizes to the nuclei of hepatocytes in chronically HCV-infected patients and core transgenic mice [25], [34], [35]. In this study, we observed a small quantity of a product with lower molecule weight when full-length HCV core gene was expressed in cultured Huh7 cells. These studies suggest that the nuclear localization or truncated form of the core protein may play an important role in chronic HCV infection. Moriishi *et al.* has reported that mature (amino acids 1–173) and more truncated (amino acids 1–151) forms of HCV core protein can bind to PA28γ in the nucleus and hence induces liver steatosis and HCC development through a PA28γ-dependent pathway in core gene-transgenic mice [11], [12], suggesting that the nuclear localization of the truncated core proteins may function as a transcriptional factor or regulator. In this study, up-regulation of miR-345 expression by mature form (amino acids 1–173) of the core protein may be also associated with its nuclear localization. Indeed, we also demonstrated that more truncated core protein (amino acids 1–153) which deletes more residues of hydrophobic C-terminal region up-regulated miR-345 expression, indicating that the up-regulation of miR-345 expression may be associated with the nuclear localization of HCV core protein. MiR-345 is down-regulated in full-length HCV genome-expressing cells as reported by Braconi *et al.* [19]. Our result was not consistent with the observation from Braconi's group, since the different expressing system and different hepatoma cells were used in the experiments. There is no detectable or little, if any, amount of truncated form of HCV core protein expression in our full-length HCV replicon-expressing system. However, truncated form of HCV core protein has been demonstrated to localize in nuclei of hepatocytes in chronically HCV-infected patients and core transgenic mice [25], [34], [35].

The article "Hepatitis C Virus Core Protein Down-Regulates p21Waf1/Cip1 and Inhibits Curcumin-Induced Apoptosis through MicroRNA-345 Targeting in Human Hepatoma Cells" was retracted in 2020. Reasons: duplicated images; unreliable results or conclusions; concerns about the data; concerns about the images.

The up-regulation of miR-345 expression by HCV core protein may be associated with the demethylation of its promoter. Tang *et al.* has demonstrated that miR-345 with a CpG island in the promoter is a methylation-sensitive microRNA and is highly induced by demethylating agent in human colorectal cancer cell lines [38]. Recently, miR-21 has been identified to indirectly down-regulate DNA methyltransferase 1 (DNMT1) expression by directly targeting human *RASGRP1* gene, a known critical regulator of the upstream Ras-MAPK pathway of DNMT1 [39]. In this study, we also determined the up-regulation of miR-21 expression in HCV core-overexpressing Huh7 and HepG2 cells (Fig. S3). The up-regulation of miR-21 expression by mature form (amino acids 1–173) of the core protein may contribute to miR-345 promoter hypomethylation. Up-regulation of miR-21 expression has been reported in HCV infectious clone-infected Huh7.5 cells and patients with chronic HCV infection [40]. In our study, the mature form (amino acids 1–173) of the core protein can enhance miR-21 expression, however, the full-length core protein had no effect on miR-21 induction. This finding suggested that the mature form (amino acids 1–173) of the core protein was relevant to the regulation of cellular microRNAs in chronic HCV infection. In fact, we also initially observed the modulation of most of cellular microRNAs by mature form (amino acids 1–173) of the core protein (Fig. 1B). Further confirmation will be needed.

Up-regulation of miR-345 expression may involve in cancer development. Some studies have described the up-regulation of miR-345 expression in human cancers including oral squamous cell carcinomas and malignant mesothelioma [41], [42]. A recent study also reveals that some tumor-related microRNAs including miR-345 are up-regulated from 28 published tumor studies by analyzing microRNA expression microarray datasets, indicating that miR-345 may be an oncomiR in human cancers including HCC [43]. MiR-345 has been reported to down-regulate *BAG3* gene expression, an anti-apoptosis gene, as a tumor suppressor microRNA in human colorectal cancer [38]. However, in our study, miR-345 down-regulates *p21^Waf1/Cip1^* gene expression as an oncomiR in human hepatoma cells. These two studies suggest that the same microRNA may function as an oncogene or as a tumor suppressor gene depending on cell types and microenvironment. Our study shows that the up-regulation of miR-345 expression may be related to hepatocarcinogenesis during chronic HCV infection.

The article "Hepatitis C Virus Core Protein Down-Regulates p21Waf1/Cip1 and Inhibits Curcumin-Induced Apoptosis through MicroRNA-345 Targeting in Human Hepatoma Cells" was retracted in 2020. Reasons: duplicated images; unreliable results or conclusions; concerns about the data; concerns about the images.

In conclusion, our study demonstrates that mature or more truncated HCV core protein (amino acids 1–173 or 1–153) can up-regulate the expression of miR-345 which then suppresses *p21^Waf1/Cip1^* gene expression in human hepatoma cells. We also show that mature HCV core-induced miR-345 can suppress endogenous *p21^Waf1/Cip1^* gene expression in HepG2 and curcumin-stimulated Huh7 cells. Furthermore, we demonstrate that mature HCV core-induced miR-345 involves in anti-apoptosis through down-regulation of *p21^Waf1/Cip1^* gene expression in curcumin-stimulated Huh7 cells. In conclusion, it is the first time that HCV core protein has ever been demonstrated to inhibit human *p21^Waf1/Cip1^* gene expression through miR-345 targeting.

## Supporting Information

Figure S1 **MicroRNA-93 cannot down-regulate endogenous** ***p21^Waf1/Cip1^*** **gene expression in human hepatoma cells.** HepG2 cells were transiently transfected with the increased amount of miR-93 mimic for 24 hours. The *p21^Waf1/Cip1^* gene expression at protein level was determined by Western blotting. β-actin served as an internal control.
(TIF)

Figure S2 **Curcumin has no effect on endogenous miR-345 expression.** Huh7 cells were treated with curcumin in dose- (left panel) and time- (right panel) dependent manners. The relative expression of miR-345 was determined by TaqMan real-time qPCR. Data was shown as the means ± S.D. from triplicate experiments. *P<0.05.
(TIF)

Figure S3 **HCV core protein up-regulates miR-21 expression in human hepatoma cells.** Huh7 and Hepg2 cells were transiently transfected with empty vector (labeled with Mock) and three HCV core gene-expressing vectors, pT-REx-HA-Core191 (labeled with HA-Core191), pT-REx-HA-Core173 (labeled with HA-Core173), and pT-REx-HA-Core153 (labeled with HA-Core153), for core protein with amino acids 1–191, 1–173 and 1–153, respectively. At 48 hours after transfection, relative expression of miR-21 was determined by TaqMan real-time qPCR in Huh7 cells (left panel) and HepG2 cells (right panel). Data was shown as the means ± S.D. from triplicate experiments. *P<0.05, **P<0.001.
(TIF)

Figure S4 **Curcumin induces apoptosis through p21^Waf1/Cip1^-independent pathway in HepG2 cells.** HepG2 cells were treated with different doses (6.25, 12.5, 25, and 50 µM) of curcumin for 24 hours. DMSO served as control (labeled with 0 µM). The *p21^Waf1/Cip1^* gene expression at protein level was determined by Western blotting (upper panel). β-actin served as an internal control. Apoptosis was determined by annexin V-FITC apoptosis assay (lower panel). Original magnifications ×200. Cells from early apoptotic stage were stained with annexin V-FITC, and appeared green. Cells from late apoptotic stage were stained with both annexin V-FITC and PI, and merged to be yellow.
(TIF)
